The article "Lung Cancer Prediction from Text Datasets Using Machine Learning" was retracted in 2023. Reasons: unreliable results or conclusions; concerns about the data; concerns about the peer review; concerns about the citations.

# Lung Cancer Prediction from Text Datasets Using Machine Learning

**DOI:** 10.1155/2022/6254177

**Published:** 2022-07-14

**Authors:** C. Anil Kumar, S. Harish, Prabha Ravi, Murthy SVN, B. P. Pradeep Kumar, V. Mohanavel, Nouf M. Alyami, S. Shanmuga Priya, Amare Kebede Asfaw

**Affiliations:** ^1^Department of Electronics and Communication Engineering, R. L. Jalappa Institute of Technology Doddaballapur, Bangalore, Karnataka 561203, India; ^2^Medical Electronics Engineering, Ramaiah Institute of Technology, Bangalore, Karnataka 560054, India; ^3^Department of Computer Science and Engineering, S J C Institute of Technology, Chikkaballapur, Karnataka 562101, India; ^4^Department of Electronics and Communication Engineering, HKBK College of Engineering, Bangalore, Karnataka 560045, India; ^5^Centre for Materials Engineering and Regenerative Medicine, Bharath Institute of Higher Education and Research, Chennai 600073, Tamil Nadu, India; ^6^Department of Mechanical Engineering, Chandigarh University, Mohali, 140413 Punjab, India; ^7^Department of Zoology, College of Science, King Saud University, PO Box 2455, Riyadh 11451, Saudi Arabia; ^8^Department of Microbiology-Immunology, Northwestern University, Feinberg School of Medicine, Chicago, IL 60611, USA; ^9^Department of Computer Science, Kombolcha Institute of Technology, Wollo University, Ethiopia

## Abstract

Lung cancer is the major cause of cancer-related death in this generation, and it is expected to remain so for the foreseeable future. It is feasible to treat lung cancer if the symptoms of the disease are detected early. It is possible to construct a sustainable prototype model for the treatment of lung cancer using the current developments in computational intelligence without negatively impacting the environment. Because it will reduce the number of resources squandered as well as the amount of work necessary to complete manual tasks, it will save both time and money. To optimise the process of detection from the lung cancer dataset, a machine learning model based on support vector machines (SVMs) was used. Using an SVM classifier, lung cancer patients are classified based on their symptoms at the same time as the Python programming language is utilised to further the model implementation. The effectiveness of our SVM model was evaluated in terms of several different criteria. Several cancer datasets from the University of California, Irvine, library were utilised to evaluate the evaluated model. As a result of the favourable findings of this research, smart cities will be able to deliver better healthcare to their citizens. Patients with lung cancer can obtain real-time treatment in a cost-effective manner with the least amount of effort and latency from any location and at any time. The proposed model was compared with the existing SVM and SMOTE methods. The proposed method gets a 98.8% of accuracy rate when comparing the existing methods.

## 1. Introduction

To put it another way, lung cancer is the leading cause of mortality in both men and women worldwide [1]. According to other studies, pulmonary cancer accounted for roughly 13% of all cancer diagnoses in the United States in 2015. Lung cancer accounts for approximately 27% of all cancer-related deaths, according to the American Cancer Society [2]. As a result, lung nodules in the early stages of development must be properly examined and monitored. Cancer development and progression were investigated by the researchers in this study using the ML and DL methodologies for predicting cancer growth and progression. The prediction models discussed here are built using a variety of supervised machine learning algorithms as well as various input and data samples. Using the image operator LBP, images can be turned into arrays or images of integer labels, which are referred to as local binary patterns. These labels are used in further image analysis, which is most typically presented in the form of a histogram. As a result of the LBP texture operator's ability to be specific and how easy it is to use, it has been used in a wide range of applications [2].

The histogram then makes use of these markers to conduct a more thorough analysis of the image. In the previous three years, cancer mortality from lung disease has remained greater than cancer mortality from prostate or breast cancer in both men and women [3]. In large part, this is owing to the sophisticated and systemic character of the prognostic models for prostate and breast cancer that have been developed in recent years. To do this, it is necessary to develop a reliable early-stage lung cancer forecast model as soon as possible [4–6]. An effective predictor in both linear and nonlinear scenarios, SVM, has found widespread use across many industries, including medicine [6–8]. Still, cancer prognostic models are being made even though SVM is a great way to classify things [9]. Patients' best treatment options are determined by the results of a mutation test [10], which has become more important in clinical trials. In addition to screening, direct sequencing can be used to uncover mutations that were missed during the screening process. A genetic mutation in the EGF receptor (EGFR) has been discovered and can be utilised to detect genetic mutations in lung cancer [10–13]. It has been demonstrated that the artificial neural network (ANN) and support vector machine (SVM) outperform their nonensemble counterparts [14]. Because the majority misjudgment carries a bigger weight than the minority, miss judgment is more likely to occur for the majority than for the minority. Classification algorithms that rely on traditional methods of doing things do not perform as well as they could [15–19].

In this paper, we optimise the process of detection in the lung cancer dataset using a machine learning model based on SVMs. Using an SVM classifier, lung cancer patients are classified based on their symptoms at the same time as the Python programming language is utilised to further the model implementation. There are various diagnostic methods for different tumours. But there are only a few specific ways to calculate what populations are in them. This paper will introduce the method of not only diagnosing cancerous tumours but also doing the work required to calculate their size, shape, and location. Thus, not only can tumours be detected but also their type can be easily identified by counting and winning and can calculate the proper guidelines for dealing with them.

## 2. Related Works

The authors [3] experimented to assess the impact of the referral course and side effects on delays in a fast outpatient indicative programme for suspected lung cancer patients, as well as to determine whether delays were associated with sickness stage and outcome. There has been a thorough examination of the characteristics of tumours, their organisation, and the many deferrals that have occurred. A total of 565 patient restoration schematics were collected for this study. In total, 51% of the participants had lung growths while the other half (8.5%) had a variety of injuries, with 111 people (19.6%) having radiological anomalies that were not regarded to be potentially life-threatening. When it came to hemoptysis, first-line wait times were much lower than in other cases. During the rule-making process, an RODP was developed to facilitate the analysis process. It is estimated that the vast majority of patient postponements are caused by deferrals in the first and second lines of treatment.

They [11] investigated several different ways of measuring lung growth. There were several of these, including the application of artificial neural networks, image processing, linear dependency analysis (LDA), and the self-organizing map (SOM). In conclusion, it is recommended that support vector machines be used as a characterization technique. When you use machine learning, you can use support vector machines to look at information and recognise patterns. At the beginning of their research, [10] devised a technique to detect lung growth. Data preprocessing is carried out in this manner to kick off the process of enhancing the photograph. When the datasets are ready for testing under information mining and neural systems, which are both crucial to distinguishing across rehabilitative methods, this is the point at which they can be tested. Using back-propagation neural networks to classify information images as either malignant or nondangerous, the researchers were able to accomplish the desired result (BPNN). People who work in medicine figure out which stage of malignancy will be most helpful to them when they make a diagnosis.

This work [20] employed network-based biomarker identification and quality set improvement strategies to find and approve characteristics linked with lung cancer progression and related pathways. They found that, in addition to the traits predicted by prior findings in these areas, the data revealed a wide range of innovative and surprising qualities with putative physiological capacities in smoking, which were not predicted by earlier findings in these areas. A network-based technique was devised by [21] to deal with observable confirmation of smoking and classifying between the qualities associated with lung tumour survival and those associated with nonsmoking groups and identifying all of the qualities associated with lung tumour survival and those associated with nonsmoking groups. It has been shown that a six-quality mark connected with smoking can predict the risk of lung expansion and the likelihood of survival. People who smoke may be able to see and identify lung growth if this quality mark is used.

They [22] employed information mining and streamlining approaches to generate findings from a large number of datasets to investigate lung growth. It can be used to find and exploit malignancy patterns in databases. These patterns, which are found in databases, can then be used to predict the outcome of an illness based on the specific therapeutic instances that have been stored in the databases. The authors [23] demonstrated the detection of neuronal system expansion using computed tomography images and a computer-aided diagnosis- (CAD-) order technique, which was previously reported. To reconstruct the lung, the highlights of the CT scans were stitched together and then rebuilt. The mean, standard deviation, skewness, and kurtosis, as well as the fifth and sixth central moments, were all used to determine malignancy in the data. To improve grouping, neural networks that feed forward and backward are used to arrange things.

There is no denying that the authors [5] have been working on the application of various artificial intelligence techniques for detecting diseases and providing medications for quite some time now [5]. An artificial neural network (ANN) can be used to analyse data about breast cancer. The data from microarrays and the UCI machine learning library can be used to detect the emergence of lung cancer using multilayer feedforward neural networks that are similar to ANNs. The back-propagation rule is utilised in the preparation of the system. Using crossapproval, datasets with varying numbers of hidden layers, and hubs connecting to the same dataset can be tested against one another. If an event from the UCI dataset (bosom tumour) occurs, it is envisaged that the precision of this framework will improve as a result of the various blends of veiled layers and connected hubs. The number of hubs and hidden layers in the NCBI dataset continues to expand, resulting in an increase in precision in the analysis. If you use a similar neural system, you can predict how a patient's condition will go. This can be done with the help of an automated decision system.

Computer-aided analysis, fuzzy-weighted preprocessing, and a counterfeit-resistant acknowledgement system were all employed in the study conducted by [24]. The framework is broken down into three stages. Although the dataset contains 57 high points, only four of these high points can be investigated using traditional component analysis. The use of a weighting approach based on the prehandling of fuzzy weighting was employed as a preparatory step before the primary classifier was implemented. Third, a classifier for counterfeit safe acknowledgement was utilised to identify the counterfeits. The lung dataset was used to evaluate a programmed approach to tumour analysis that was developed by the researchers. It was very encouraging for grouping applications in the future to see that the framework characterization was 100% correct, which was a very good news.

According to [25], an emotion-aware recommender system that is based on the integration of user via social network data, explicit rating data, and sentiment data derived from user reviews can be utilised to produce suggestions [26]. With the help of this technology, it is possible to improve the accuracy of prediction ratings and suggestions. The authors [26] developed reliable prediction systems for nonstop capacity which is reduced. While this technology does not provide as much productivity as classic higher-order feedforward systems, it does provide a more consistent and productive design while preserving its quick learning qualities. The pi-sigma organisation hypothesised that they will utilise a rare form of edge polynomial in their edge polynomial system, which is a rare type of edge polynomial. The capability of any multivariate polynomial to be addressed by an RPN in this frame and acknowledged as an RPN response is demonstrated in this frame. The incremental system development process is given a particular systemic framework through the use of RPN. According to the evidence, there appears to be an efficient computation for the system that results in smooth speculation and continual learning.

A method for predicting lung disease, recognising it early, and treating it while the lung tumour is still small has been discovered by [27]. To better prepare for the lung disease, certain highlights were removed from the photographs. It has been discovered that the design of acknowledgement-based systems has an impact on the ability to anticipate pulmonary development. When it came to doing a full examination of previous experience with lung tumour demands, image handling procedures were employed. Computer-based image-preparation tools can be used to predict and control lung expansion, and they can help you do this.

According to [28], non-small-cell lung cancer can be reliably predicted using a new approach that can recognise financially smart biological signals in the body (NSCLC). The complexity of tumours means that one can only make educated guesses regarding their current state by integrating several factors. The study collection of 12,600 quality-profiled NSCLC articulation profiles revealed the presence of nine quality marks that can be utilised to diagnose NSCLC lung carcinoma and to identify familial markers for the disease. The researchers used an approach in which they used a modest and already obscure arrangement of organic markers to achieve an idealised prediction precision (99.75%) for diagnosing the illness of a subtype of disease to discover genetic markers for NSCLC subtypes.

The MLPNN algorithm was used to analyse the components of the lung CT images, and the crossover hereditary and molecular swarm improvement techniques were proposed in [29]. It was found to be a reliable source of information when compared to lung CT scans. Using guided visuals to calm down agitation was associated with better extraction results, and preprocessed images were employed to aid in the extraction process. We were able to extract these highlights with the use of the MAD approach. Individual highlights were selected with the help of GAPSO. The final image result is generated using the GAPSO-MLPNN algorithm. As a starting point, it turns out that a large range of test data has outstanding geometric precision, high classification accuracy, and low bit error rates, and this is true across the board. In addition to its outstanding performance, this technology can identify lung illnesses.

They [30] employed a back-propagation neural network to construct a model for forecasting the price of commodities. The author next proposes a self-evolving trading strategy that conforms with the rules of the futures trading market, the data from the testing. Finally, the new tactics are compared to the traditional techniques to demonstrate how their strategy has evolved overtime. Experiments have revealed that his answers surpass those of the other researchers for the proposed assessment indicator. His strategy outperforms the competition in terms of both yield and risk. According to [31], hybrid feature extraction and, as a result, improving the stability of authentication of the ECG data was proposed. Additional development was the creation of a parallel pattern recognition framework for ECGs, which improved the efficiency of recognition across diverse ECG feature spaces. After the tests were done, it was found that the authentication method that was suggested is good.

The authors of [32] have presented a hybrid system, which they have tested on authentic SinaWeibo datasets. People who looked at the results say that the new hybrid recommendation algorithm is better than its predecessors in terms of performance and has a better performance than other algorithms. The details of the existing machine learning models used in the study is illustrated in Figure 1.

## 3. Proposed Method

In this section, an SVM classifier helps in the classification of lung cancer patients based on their symptoms. Preprocessing takes place before data collection in the methodology that has been proposed. With the use of a traditional 10-fold crossvalidation procedure, the selected classifiers are next trained and evaluated on the benchmark dataset for the second time. The data is calculated and evaluated to determine the most effective method of detecting lung cancer.  Figure 2 represents an overview of the planned strategy at the highest level.

All the data given first are given as input in order. The different types of data on which these inputs are based also require the required information of the data from different volumes to be subjected to a large number of different analyses and extracted based on its results. These preprocess methods convert the input data into the required small groups and process them accordingly. Data for this processing process are classified into separate groups. In these segmentation operations, the basic form size of the dataset and the rate of operation is calculated and classified. After finally classifying them, the applications of its toddlers are extracted.

### 3.1. Data Acquisition

For this investigation, we used a dataset from the University of California, Irvine, online repository named Lung Cancer. The dataset comprises a total of 32 instances, 57 characteristics, and one class attribute in its entirety. The fundamental purpose of our proposed study is to evaluate and compare the performances of SVM, among others.

### 3.2. Data Preprocessing

Preprocessing is the initial step in the detection of lung cancer, and it entails filling in any gaps in the dataset and deleting any information that is not strictly necessary. As a result, missing values are imputed using the *K* nearest neighbour approach with three neighbours to increase the overall reliability of the entire dataset. Both training and testing samples are required.

### 3.3. Training and Testing Samples

The input data samples are first trained and then tested using a neural network, which is a type of artificial intelligence. The weights of the neural network are determined at random from the input data at the beginning of the process. The neural networks are trained on a sample dataset, and they are then evaluated on the same dataset that was used for training. During the classification process, data is weighed to ascertain the frequency of errors or error rates that occur, and the errors are repaired by reweighting the dataset.

### 3.4. Feature Extraction

For a large number of features to be extracted from a dataset to lessen the complexity of detecting lung cancer, the dataset must be segmented. This detecting technology will remove the tumour from the lung that has developed as a result of the multiplication of cancer cells (features). This feature extraction approach makes use of the PSO programming language. Feature extraction from input data is a component of pattern recognition algorithms, and it is used to obtain the main qualities that are more useful and nonredundant, as well as collect cancer-related information to anticipate patient circumstances for interpretation, using SVMs to categorise data.

### 3.5. Classification Using SVM

Classification is the process of organising information into logical groups. Decisions can be made on the basis of both structured and unstructured data, which can be analysed by the system. Malware and denial-of-service (DoS) attacks can both be prevented and mitigated by using data mining techniques. This means that texts are automatically edited and categorised to make sure that their integrity is kept at all times.

In addition to the standard classifications of cancer as either malignant (M) or benign (B), a new classification named premalignant has been added to the B. Patients that fall into this category will receive an increased level of attention and treatment alternatives. When it comes to data security, categories such as copied, sent, and retrieved data will always be on the lookout for suspicious activity. The practise of providing meaningful labels to data in order to increase its usability and discoverability is known as classification. By reducing redundant data, it can help you save money on storage and backup costs. As a result, processing times can be significantly shortened in some cases.

In order to discriminate between items belonging to different classes, the SVM is an algorithm that trains machines to learn on their own with the aim of discriminating between them. Given that the margin of a hyperplane is determined by the instance that is closest to it, an optimal SVM model would comprise hyperplanes that split classes as widely as possible.

The SVM primary goal is to maximise profit margins as much as possible. Given the training dataset *x*_*i*_ and a feature vector of dimension *n*, the classification is given by *y*_*i*_ ∈ {−1, 1}, where *i* = 1, ⋯, *N* with training data *N*, and the classification is carried out.

When constructing a linear classifier, Equation (1) makes use of the hyperplane normal weight vector *ω*, which is defined as rescaled hyperplane classifiers that satisfy Equation (2), and the weight vector is determined by subtracting the rescaled weight vector from the original weight vector as in Equation (3).

It is possible to solve Equation (3) using the Lagrange function in Equation (4), which results in the values of *ω* = ∑_*i*_*α*_*i*_*y*_*i*_*x*_*i*_ and *b* = *y*_*i*_ − *ω*^*T*^*x*_*i*_ as a result of the solution. It is used to denote the Lagrange multipliers for each inequality constraint, which stands for inequality constraint multipliers.

(1) $$\begin{array}{c} f\left(x\right)=\mathrm{sign}\left(\omega x+b\right), \end{array}$$

(2) $$\begin{array}{c} y_{i}\left(\omega^{T}x_{i}+b\right)\geq 1,i=1,\cdots ,N, \end{array}$$

(3) $$\begin{array}{c} \text{minimize }\frac{1}{2}\omega^{T}\omega s.t.y_{i}\left(\omega^{T}x_{i}+b\right)\leq 1,i=1,\cdots ,N, \end{array}$$

(4) $$\begin{array}{c} L\left(\omega ,b,\alpha \right)=\frac{1}{2}\omega^{T}\omega +\underset{i}{\sum }\alpha_{i}\left(1-y_{i}\left(\omega^{T}x_{i}+b\right)\right). \end{array}$$

Because nonseparable data cannot be separated, Equation (2) is altered to Equation (3) by including a slack variable *ξ* as in Equation (5). This is achieved by multiplying the 0.5 *ω*^*T*^*ω* by a penalty constant *C*, yielding Equation (6). A misclassification of a training example can result in a penalty constant *C* being applied to your account. For lower values of *C*, the optimization will select a hyperplane with a large margin of safety, which may result in a greater number of points being wrongly classified.

In practice, a wide range of values for parameter *C* is usually utilised, and the optimal performance is evaluated using a separate validation set or by crossvalidation to check the performance using only one training set, depending on which method is preferred.

(5) $$\begin{array}{c} y_{i}\left(\omega^{T}x_{i}+b\right)\geq 1-\xi_{i},i=1,\cdots ,N, \end{array}$$

(6) $$\begin{array}{c} \text{minimize }\frac{1}{2}\omega^{T}\omega +C\xi_{i}s.t.y_{i}\left(\omega^{T}x_{i}+b\right)\leq 1-\xi_{i},i=1,\cdots ,N. \end{array}$$

When used in conjunction with kernel functions, a linear hyperplane can be utilised to separate support vectors that are not linearly separable. Nonlinear SVM classifiers that are nonlinear in nature frequently use the radial basis function (RBF) kernel as their kernel function. We can infer this from the feature map *ϕ*(*x*), which is *K*(*x*_*i*_, *x*_*j*_) = *ϕ*(*x*_*i*_)^*T*^*ϕ*(*x*_*j*_).

In the following Equation (7), we see the RBF kernel. We use the formula *γ* = 1/2*σ*^2^ to reduce the number of terms in the equation. The Lagrange function may be used to produce Equation (8), where *α* is the solution to the dual problem in Equation (7), which is the solution to the dual problem in Equation (9). We can now relax (10), having finally arrived at the conclusion predicted by Equation (10).

(7) $$\begin{array}{c} K\left(x_{i},x_{j}\right)=\exp\left(-\frac{{\left\|x_{i}-x_{j}\right\|}^{2}}{2\sigma^{2}}\right)=\exp\left(-\gamma {\left\|x_{i}-x_{j}\right\|}^{2}\right), \end{array}$$

(8) $$\begin{array}{c} b=y_{i}-\underset{j}{\sum }\alpha_{j}y_{j}K\left(x_{j},x_{i}\right)\forall i∙\alpha_{i}>0, \end{array}$$

(9) $$\begin{array}{c} \underset{i}{\sum }\alpha_{i}-\frac{1}{2}\underset{i,j}{\sum }\alpha_{i}\alpha_{j}y_{i}y_{j}K\left(x_{i},x_{j}\right),\text{s}.\text{t}.\underset{i}{\sum }\alpha_{i}y_{i}=0, \end{array}$$

(10) $$\begin{array}{c} \omega^{T}x+b=\underset{i}{\sum }\alpha_{i}y_{i}K\left(x_{i},x\right)+b. \end{array}$$

When it comes to binary classification problems, it is a usual practise to employ the SVM approach to solve them. A one versus one strategy is proposed in which a binary model is generated for each of the predicted classes, and a prediction is made based on the binary model confidence measure on that class when compared to all of the other classes.

## 4. Results and Discussions

The data was located in the machine learning repository at UCI, and there are 32 examples in the dataset, each having 57 features and a notional range of 0-3 for all predictive attributes. This is accomplished by translating nominal attribute and class label data into binary form, which makes data analysis easier to perform. The conversion of data from nominal to binary form is the most widely used and standardised method in data analysis. There are some missing values in the dataset, which has an impact on the performance of the algorithm; therefore, caution should be exercised when analysing the data. The label has three different levels of severity: high, medium, and low. There is a significant amount of missing data in the input data. As a result, it is important to prepare the data in such a way that the missing values are replaced with the value that occurs the most frequently in the column. Following that, the newly processed data is subjected to analysis using a Python tool. When prior data is transformed into a form that may be utilised for categorization, classifiers are used to do this. To put the classifier through its paces, ten different crossvalidation methods are applied. It is a powerful data analysis approach that can be used to run ten times the number of computations with the available data and create accurate predictions based on that data as is possible with traditional methods. The classification accuracy of a forecast is defined as the number of correct predictions produced out of a total forecast. The values of these variables are conditional on the outcome of the experiment. In the case of false-positive and false-negative values, they are denoted by the true positive (TP) and true negative (TN). As you can see, false positive (FP) and stands for false negative (FN).

The method proposed is the most efficient method. This is because of the computations that exist in this system. That is, after the given data is included, many of the data in the fifth text are compared with its various formats and analyzed. These analysis methods compute its structure and dimensions when comparing the given data with the many data present in the other datasets attached to it. The various data available in such calculations will define its boundaries. The changes in its boundaries when small cooks are attached to each other help to calculate it more accurately when analyzing its various shape models. Thus, its accuracy is high.

As demonstrated by the evaluation findings, SVM with SMOTE resampling (Figures 3–8) on two iterations of the Lung Cancer dataset produced the greatest performance on the dataset. When compared to earlier methods, this method achieves the maximum value for all of the parameters that were investigated. The study has two minorities participating in our lung cancer data collection. As a result, after two rounds of SMOTE, there is an equal distribution of minorities among the two classes. The third run of SMOTE generates synthetic samples for class B, which had previously been the majority class in the previous steps. Nonetheless, the classification performance of these samples does not increase. The best way to use SVM and SMOTE is to do both of them twice on the same dataset.

Effectiveness is defined as the ability of a machine learning model to outperform other models that are currently available. It was decided to use lung cancer data to compare the proposed heuristic classification strategy to other current classification methods, including neural networks, decision trees, and regression analysis, in order to determine which was superior. When comparing the accuracy of the KNN method against that of the decision tree classifier, the KNN algorithm came in at 68.9%. Overfitting and variance have been reduced as a result of the random forest with embedded attribute optimization feature, which has resulted in an increase in classification accuracy. The model training phase provides you with the option of selecting qualities from a list of predefined attributes. When SVM and SMOTE are used together, the attribute set is further optimised, and the accuracy is improved even further. The proposed model had a 98.8% accuracy rate.

To assess the model performance, a range of cancer datasets were employed to assess its performance. In order to limit the number of features available, all cancer datasets were taken into consideration. A random forest classifier was used in conjunction with a proposed technique, which resulted in enhanced classification accuracy.

Performance metrics such as *f*-measure and specificity were also used to assess the overall effectiveness of the proposed hybrid heuristic classifier model in a variety of ways, including classification accuracy. A total of five cancer datasets were analysed for this study. Overall, the proposed heuristic-based classification technique resulted in a classification result that was reasonably consistent.

## 5. Conclusions

Predicting lung cancer is one of the most challenging medical challenges to address due to the complexity of cancer cells. In addition to lung cancer, there are over 100 other types of cancer to be concerned about. If treatment for lung cancer is delayed, there is a significant increase in the risk of death. If cancer is detected and treated early enough, it is possible to cure it. In this work, SVM is used to predict the development of lung cancer. The fundamental objective of this system is to provide consumers with an early warning, allowing them to save both money and time. The performance evaluation of the proposed method produced positive results, demonstrating that SVM can be used effectively by oncologists to aid in the identification of lung cancer. If the prediction is right, it is possible that the doctor will be able to prepare a better prescription and present the patient with an earlier diagnosis.

## Figures and Tables

**Figure 1:** Conventional machine learning models.

**Figure 2:** Proposed design.

**Figure 3:** Accuracy.

**Figure 4:** Precision.

**Figure 5:** Recall.

**Figure 6:** *F*-measure.

**Figure 7:** Correctly classified.

**Figure 8:** Incorrectly classified.

## Data Availability

The data used to support the findings of this study are included within the article. Further data or information is available from the corresponding author upon request.
